The article "A Risk Decision-Making Model Based on Kalman Filter for Intellectual Property Pledge Financing" was published in 2022. Journal: Comput Intell Neurosci.

# A Risk Decision-Making Model Based on Kalman Filter for Intellectual Property Pledge Financing

**DOI:** 10.1155/2022/8025455

**Published:** 2022-02-27

**Authors:** Xianan Yin, Hua Ming, Xinzhong Bao

**Affiliations:** Management College, Beijing Union University, Beijing 100101, China

## Abstract

Risk dynamic early warning is of great importance for financing risk decision-making. Intellectual property (IP) pledge financing is an effective way to alleviate the financial difficulties for technologically small- and medium-sized enterprises (SMEs). It is very important to study the financing risk decision-making because of its higher risk compared with other mortgage loans. Based on Kalman filter, we establish the pledge financing risk decision-making model and extract the key variables affecting financing risk by principal component analysis. We test the model with 88 listed SMEs. The results show that the average error between the predicted and the real values is 8.5% and the overall recognition accuracy of the model is 89.1%. The risk decision-making model has high discriminant accuracy and can provide evidence to risk decision-making.

## 1. Introduction

Technology SMEs are counted as one of the most technologically advanced enterprises that assign great large amount of money to their development [1, 2]. Furthermore, intellectual property pledge financing is an effective way to alleviate the financing difficulties of technology SMEs. As the significant differences between IP pledges and traditional physical pledges lead to specificity in both asset valuation risk and disposal risk, risk is a primary consideration when stakeholders make financing decisions. However, the risk is an uncertain event or condition that, if it occurs, has a negative effect, and it could happen at any stage without warning [3]. Therefore, many scholars have studied the IP pledge financing risks in different aspects. Pennington & Sanchez (2007) and Crawford & Strasser (2008) studied the IP pledge financing risks in different stages from three dimensions: credit risk, infringement risk, and compensation risk [4, 5]. Moreover, from the essence of IP pledge financing risk, in addition to the quality of the pledged goods, the stakeholders of pledge financing pay more attention to the financial and operational conditions of the financing enterprises. Liu Peipei (2011) believes that the risk of IP pledge financing depends on the value of the pledged goods formally, but on the overall business capacity of enterprises essentially [6], which has also been shared by most scholars. While the financial status and operating conditions of an enterprise are a dynamic process that develops and changes in real time, a dynamic risk decision model could better characterize the risk of IP pledge financing.

The article "A Risk Decision-Making Model Based on Kalman Filter for Intellectual Property Pledge Financing" was published in 2022. Journal: Comput Intell Neurosci.

The current research on the risk of IP pledge financing mainly focuses on the construction of a financing risk index system [7–9], while the research on financing risk decisions is limited to static evaluation and analysis. In addition, an advanced tool for validating decisions is necessary to ensure the smooth operation of corporate activities [10]. Although common methods can be used to evaluate financing risks, including factor analysis method [11], VIKOR method [12], interval number TOPSIS [13], hierarchical analysis method, and fuzzy comprehensive evaluation method [14], they mainly use the cross-sectional data, which cannot reflect the cumulative formation process of risks, so the models of traditional methods are not stable enough, which reduces the accuracy of risk decision-making. Besides, decision-making action that effectively extracts and utilizes enough data about decision based on big data is a trend [15].

In order to improve the effectiveness of risk decision-making, scholars have tried to introduce a dynamic risk decision model called BP neural network that calculates the error between the calculated output value and the true value, and continuously adjust it until the acceptable error level [16, 17]. Zeng and Ming evaluate the risk of IP pledged financing for technology-based SMEs empirically [18]. BP neural network achieves early warning of dynamic risk with the deep learning algorithms, but it is essentially an approximation algorithm for linear weight functions, which is more effective if there is no correlation among processing data. As for the strong correlation of time series data of business operations, it would reduce the effectiveness of early warning of dynamic risk. Therefore, IP pledge financing risk requires methods that can analyze data with correlated time series and reflect the risk formation process, and Kalman filtering meets these needs well. Compared with other methods, the Kalman filter has two advantages. First, the correlation among processing data will not affect the results. Second, the filtering process is an acyclic recursive process of automatically updating “prediction-correction” with the latest data, and it does not need to save the historical measurement data. The enterprise's IP pledge financing risk is a dynamic state with enterprise operation, and the previous risk will affect the status of the next period state. Therefore, the Kalman filtering method can predict the dynamic financing risk and determine the level of financing risk.

Kalman filtering has been widely used in the field of management for monitoring risk [19], especially for dynamic risk. Sun et al. established a Kalman filter dynamic early-warning model for financial crises, and the results showed that Kalman filter-based dynamic model is more accurate than other prediction models [20]. Zhu studied the financial crises in different life cycle stages of enterprises based on the dynamic model of Kalman filter combined with the logistic regression method [21]. Fu et al. constructed an early-warning model of financial risk with the fusion of neural network and Kalman filter and verified that enterprise financial index data has a good predictive effect on the enterprise financial risk [22].

The article "A Risk Decision-Making Model Based on Kalman Filter for Intellectual Property Pledge Financing" was published in 2022. Journal: Comput Intell Neurosci.

In summary, the Kalman filter theory is more applied to the dynamic early warning of enterprise financial risk, not to the financing risk decision-making. Since the Kalman filter can describe the cumulative process of risk change and provide risk early warning by the time series data, we will try to establish a financing risk decision-making model based on Kalman filter and test the accuracy and effectiveness of the model.

The possible contributions of this paper are mainly reflected in two aspects: (1) We construct a dynamic decision-making model instead of the previous static model, which improves the accuracy of risk decision. (2) We introduce a risk decision-making method which is not affected by time series correlation data. The Kalman filtering method could eliminate the adverse effects of the correlation data. According to the dynamics and accumulation of financing risk, we use the self-cyclic recursive characteristics of Kalman filter to identify the parameters of the model and estimate the risk status with the time series financial data, and visualize the financing risk level.

## 2. A Risk Dynamic Decision-Making Model

### 2.1. Kalman Filtering

Kalman filter is a method based on state-space model, which can estimate the hidden state of the system in real time through the observation with noise, so as to solve the problem of state-space estimation. The method can also include any number of unknowns; it treats the signal process as the output of a linear system under the action of white noise and uses the state equation to describe this input-output relationship, using the statistical properties of the system state equation, the observation equation, and the white noise excitation (system noise and observation noise) to form a filter with recursive characteristics algorithm. The core consists of the following five equations:

State updating equation: the state estimation of the current time point from the previous state is as follows:

(1) $$\begin{array}{c} {\hat{x}}_{t}=A_{t}{\hat{x}}_{t-1}+u_{t}. \end{array}$$

The calculation of the estimated covariance of the current time point state is as follows:

(2) $$\begin{array}{c} P_{t}^{-}=A_{t}P_{t-1}A_{t}^{T}+Q_{t}. \end{array}$$

Measuring updating equation: the calculation of Kalman gain is as follows:

(3) $$\begin{array}{c} K_{t}=\frac{P_{t}^{-}H_{t}^{T}}{H_{t}P_{t}^{-}H_{t}^{T}+R_{t}}. \end{array}$$

*y_t_* i, smeasured to update the state estimation.

(4) $$\begin{array}{c} {\hat{x}}_{t}={\hat{x}}_{t}^{-}+K\left(y_{t}-H_{t}\hat{x}\bar{t}\right). \end{array}$$

Updating error covariance is as follows:

(5) $$\begin{array}{c} P_{t}=\left(I-K_{t}H_{t}\right)P_{t}^{-}. \end{array}$$

The state update equation estimates the state of the current time point using the estimated value obtained from the previous time point and the covariance of the error to obtain a priori estimate. On the other hand, the measurement update equation combines the obtained a priori estimate with the measured value to obtain an improved a posteriori estimate, which serves as feedback to the state update equation and continues to estimate the next time point. Thus, a recursive process of “prediction-correction” is formed. Among them, Kalman gain plays a role in adjusting the weight between the observed value and the predicted value, so as to make the posterior estimate closer to the real value.

The article "A Risk Decision-Making Model Based on Kalman Filter for Intellectual Property Pledge Financing" was published in 2022. Journal: Comput Intell Neurosci.

### 2.2. Establishing State-Space Model for Risk Decision-Making

In this equation, *X*_*t*_ is composed of random variables *x*_*t*_, representing the financing risk status of financing enterprises in the period, and *Y*_*t*_ is composed of observation values of various specific indicators *y*_*t*_, representing the principal component data after indicator-specific data processing. Assuming that the operating conditions of financing enterprises in each year are regarded as a discrete control process system and their real operating conditions cannot be observed, but can be predicted by the relationship between the observed values and white noise incentives, the state-space model of dynamic early warning of financing risks can be expressed by the following state equation and observation equation, respectively:

(6) $$\begin{array}{c} x_{t}=A_{t}x_{t-1}+B_{t}u, \end{array}$$

(7) $$\begin{array}{c} y_{t}=H_{t}x_{t}+v. \end{array}$$

The parameter vector *A*_*t*_ is estimated according to the historical data of the operation status of the financing enterprises. The parameter *H* used to measure the system is the value of the measurement index of the financing risk of the enterprises and corresponds directly to the output results. *u*_*t*_ and *v*_*t*_ represent the process noise and the measurement noise of the system, respectively, being a white noise sequence:

(8) $$\begin{array}{c} u_{t}∼N\left(0,Q_{t}\right), \end{array}$$

(9) $$\begin{array}{c} v_{t}∼N\left(0,R_{t}\right). \end{array}$$

The spatial state model of pledge financing risk is a single model and single measurement, and with the advance of filtering, it has convergence, so the initial value is set to 0. This dynamic early-warning model of IP pledge financing risk based on Kalman filter is constructed by time series data as the following equations.

(10) $$\begin{array}{c} Y_{t}=\left(\mathrm{11}\right)X_{t}, \end{array}$$

(11) $$\begin{array}{c} X_{t}=\left(\begin{array}{cc} 1 & 0\\ 0 & A \end{array}\right)X_{t-1}+\left(\begin{array}{c} u_{t}\\ v_{t} \end{array}\right),\left(\begin{array}{c} u_{t}\\ v_{t} \end{array}\right)∼N\left(0,H\right)\text{.} \end{array}$$

*A* and *H* will be updated continuously with the promotion of the financial data filtering of the test samples in the equations.

The article "A Risk Decision-Making Model Based on Kalman Filter for Intellectual Property Pledge Financing" was published in 2022. Journal: Comput Intell Neurosci.

## 3. Methodology

### 3.1. Data

According to the characteristics of the IP pledge financing enterprises that have been obtained from the official website of the State Intellectual Property Office in China, it can be seen that most of the IP pledge financing enterprises are small- and medium-sized technological enterprises. Accordingly, we choose the listed companies of technological SMEs as samples and exclude the following: (1) ST and *∗*ST enterprises, which have unrepresentative debt repayment ability and abnormal financial data; (2) financial insurance enterprises; (3) enterprises with incomplete data disclosure. Combining the requirements of Kalman filtering and the characteristics of loan repayment risk, this paper uses net profit and net operating cash flow as two indicators to measure the degree of financing risk of enterprises, and 88 sample enterprises are selected. The less the interval data of Kalman filtering model, the better the filtering effect, so quarterly and semiannual reports should be the appropriate data for empirical analysis. However, because of the lack of quarterly data, we use the financial data of semiannual reports from 2013 to 2016. Data mainly comes from the WIND database, and individual index data is obtained by searching the financial reports of listed companies.

### 3.2. Constructing Early-Warning Index System of Dynamic Risk

The IP pledge financing risk is mainly reflected in the financial risk and operational risk of enterprises. The influence of nonfinancial information in the operation status of enterprises will be concentrated on the financial indicators of enterprises which contain a lot of information and can be used to predict the operation status of enterprises [23]. There are obvious differences in the financial indicators between the enterprises with financial crisis and enterprises with health financial position [24]. Before the company's financial crisis begins to worsen, the relevant characteristics will be reflected in financial indicators in advance [25]. Whether the financial indicators are calculated directly or indirectly through financial reports, they can be used effectively to study the financial risk [26]. Therefore, following the principles of scientificity, comparability, and data availability, we added the indicators of cash flow and innovation ability on the basis of traditional financial risk measurement dimensions of solvency, profitability, operation ability, and growth ability to test the risk of IP pledge financing. As shown in Table 1, a risk early-warning evaluation index system of pledge financing with 21 indicators in 6 dimensions is constructed.

The article "A Risk Decision-Making Model Based on Kalman Filter for Intellectual Property Pledge Financing" was published in 2022. Journal: Comput Intell Neurosci.

### 3.3. Global Principal Component Analysis of Dynamic Data

We obtained 616 sets of multidimensional time series stereo data from 88 families in 7 periods. In order to quickly extract important information from the stereo data table and analyze the dynamic law of the system, the global principal component analysis method was used to reduce the dimension of indicators, and several interrelated numerical indicators were transformed into a few independent comprehensive indicators; that is, fewer indicators are used instead of multiple indicators to combine most of the original information. We used the global principal component method to analyze the three-dimensional data table by SPSS 20.0. The total variance and coefficient matrix are shown in Tables 2 and 3.

In order to obtain the most orthogonal principal component factors while retaining most of the information and to get the optimal input database, the first 15 global principal component factors were extracted. The cumulative contribution rate reached more than 94%, which means the effect was good. These global principal component factors are all represented by a linear combination of 21 financial indicators. According to the coefficient matrix, the formula of each principal component is shown as

(12) $$\begin{array}{c} F_{n}=\alpha_{1}x_{1}+\alpha_{2}x_{2}+\alpha_{3}x_{3}+\cdots +\alpha_{20}x_{20}+\alpha_{21}x_{21}. \end{array}$$

Among them, *n* is the number of extracted principal components (*n*=1,2,3 ⋯ 15), *α* is the coefficients of each evaluation index, and *x* refers to the standardized values of each evaluation index.

For example, the values for each of the sample companies in period *F*_1_ can be expressed as

(13) $$\begin{array}{c} F_{1}=0.53x_{1}+0.546x_{2}-0.676x_{3}+0.515x_{4}+0.186x_{5}-0.032x_{6}\\ +0.339x_{7}+0.078x_{8}+0.7x_{9}+0.808x_{10}+0.844x_{11}+0.506x_{12}\\ +0.425x_{13}+0.196x_{14}+0.215x_{15}-0.142x_{16}-0.002x_{17}+0.084x_{18}\\ +0.29x_{19}+0.43x_{20}+0.301x_{21}. \end{array}$$

The value of *F* means that the financing risk was represented by 15 principal components instead of 21 original evaluation indicators, and the interpretation rate can reach 94%. Due to the space constraints, we only listed the formula of *F*_1_ as sample. The result data will be used for the next filtering calculation.

The article "A Risk Decision-Making Model Based on Kalman Filter for Intellectual Property Pledge Financing" was published in 2022. Journal: Comput Intell Neurosci.

## 4. Results

### 4.1. Dividing Risk Level

Although the risk of IP pledge financing is an asymptotic dynamic process of the enterprise's financial situation from good to bad, the degree of risk of IP pledge financing is different at the early-warning level. Generally speaking, the most serious degree of financial risk is bankruptcy due to insolvency, while the most serious degree of IP pledge financing risk is the lack of enough cash to repay the financing money due, but far from liquidation bankruptcy. Therefore, besides the net profit, the most important factor in measuring the risk of pledge financing is adequacy of cash flow. Consequently, in this paper, we defined the degree of risk of IP pledge financing from two indicators: net profit and net operating cash flow. The specific level of risk is divided according to the following standards:

Healthy enterprises: If the net profit and net operating cash flow of enterprises are both positive during the investigation period and show an increasing trend, the enterprises are identified as healthy ones. There are 44 healthy enterprises in the 88 samples, of which 28 are forecast samples and 16 are test samples.

Mild-risk enterprises: If the net cash flow of enterprises is negative at the end of the inspection period, the net cash flow is positive at T-1 and T-2 periods, and the net profit of any period is negative during the inspection period, the enterprises are identified as mild-risk ones. There are 24 mild-risk enterprises in the 88 samples, of which 16 are forecast samples and 8 are test samples.

High-risk enterprises: According to the data of listed companies on SME technology boards, only 11 of the 75 samples with negative net operating cash flow in three consecutive periods have positive net operating cash flow in 2015. That is, if an enterprise has negative net cash flows in periods T and T-1, it has an 85% probability of negative net cash flows in period T-2, which shows that the net operating cash flow has certain sustainability. Therefore, we identified the degree of high risk which is the negative value of net operating cash flow and twice the negative value of net profit in three consecutive periods. There are high-risk 20 enterprises among the 88 samples, of which 12 are forecast samples and 8 are test samples.

The article "A Risk Decision-Making Model Based on Kalman Filter for Intellectual Property Pledge Financing" was published in 2022. Journal: Comput Intell Neurosci.

In summary, the 88 sample companies are divided into two groups: the first group is the forecast sample group, which consists of 56 companies, including 28 healthy companies and 28 risky companies, and the second group is the test sample group, which consists of 32 companies, including 16 healthy companies and 16 risky companies. Predictive samples are used as training sets to optimize the model, and test samples as detection sets to verify the effectiveness of risk decision-making model.

### 4.2. Defining Risk-Level Threshold

In this study, statistical analysis was used to extract judgment thresholds for the risky companies based on the data from the forecast sample. With a 95% confidence probability and a confidence coefficient of 1.6449, a mean value of 0.056 and a standard deviation of 0.016 were calculated for the risky sample. The lower confidence limit for a crisis in the risky sample of companies is as follows:

(14) $$\begin{array}{c} \text{down}=\text{mean}-\text{alpha}\times \text{Stanard Deviation}=0.056-1.6449\times 0.016=0.030. \end{array}$$

Similarly, under the precondition of 95% confidence probability, the confidence coefficient is 1.6449, the mean value of the calculated state for healthy samples is 0.063, and the standard deviation is 0.007. The upper confidence limit for healthy sample companies in crisis is as follows:

(15) $$\begin{array}{c} \text{up}=\text{mean}+\text{alpha}\times \text{Standard Deviation}=0.063+1.6449\times 0.007=0.075 \end{array}$$

According to the above results, the lower confidence limit is 0.030, and the upper confidence limit is 0.075. That is, when the predicted value of financing risk is less than 0.030, the high financing risk probably happens; when the predicted value of financing risk is greater than 0.075, the financing enterprises are in a healthy state; and when the predicted value of financing risk is between 0.030 and 0.075, the financing enterprises are likely to be in a state of mild financing risk.

### 4.3. Testing the Dynamic Risk Decision-Making Result

According to the global principal component analysis, we have obtained 15 principal components' factor loads and constructed a comprehensive index of the company's financial situation in each period from the characteristic value *F* and contribution rate *β* (Table 2), which is the linear combination of each principal component. We have obtained a general index *X*_*t*_ reflecting the financing risk status of each half year of the test sample, and the results are shown in Table 4.

(16) $$\begin{array}{c} Z=\beta_{1}F_{1}+\beta_{2}F_{2}+\beta_{3}F_{3}+\cdots +\beta_{14}F_{14}+\beta_{15}F_{15}. \end{array}$$

Inputting the data of 32 test samples from 7 periods into the Kalman filtering model, we obtained the predicted values of each year. The results of some samples are shown in Table 4.

The article "A Risk Decision-Making Model Based on Kalman Filter for Intellectual Property Pledge Financing" was published in 2022. Journal: Comput Intell Neurosci.

Due to the space constraints, we choose four enterprises' dynamic forecasting charts of financing risk, including two healthy enterprises and two risky enterprises, in Figure 1.

### 4.4. Result Analysis

The results of Table 4 and Figure 1 show that the dynamic pledge financing risk decision-making model based on Kalman filter is a recursive updating process. After the initial estimation of the formation state, the initial estimation is modified by inputting the updated data information every year, and the stable state of the predicted value and the real value is gradually achieved. The model is based on the cumulative deviation of the financial situation of an enterprise over time to represent the evolution process of the financing risk of an enterprise. In a certain period of time, the financial situation of a healthy enterprise is basically in a good category, and the trend of change is gradually better, but it does not exclude a temporary weakening state. The financing risk of a risky company is gradually getting worse from mild crisis to severe crisis. There are significant dynamic early-warning characteristics to predict the financing risk by cumulative variation rather than a cross-sectional state. In addition, we can determine whether the financing risk is temporary crisis or continuous deterioration in the shape of the forecast chart and observe the change point of the financing risk state, so as to realize the visual effect of financing risk decision-making. Next, we choose one of the healthy samples and risky samples to illustrate the forecast chart.

We take Yunnan Luoping Zinc & Electricity Co., Ltd. (stock code: 002114) as an example of a healthy enterprise. The enterprise was founded in 2000 and is a high-tech enterprise. Its main business is lead-zinc ore mining, zinc smelting, hydroelectric power generation, and comprehensive utilization of resources. It also has an integrated industrial chain of “mine-electricity-smelting.” At present, it has successfully developed a number of advanced production technologies for comprehensive utilization of resources, such as germanium-indium extraction, purification of workshop slag treatment, leaching slag flotation of silver, and zinc powder mill pulverizing process transformation. From the forecast chart, only the sixth observation period is slightly lower than the healthy threshold, while other observation periods are above the healthy threshold, indicating that the company's overall solvency is strong. The annual value in 2015 is much lower than that in 2014 for the reason that in the second half of 2015, due to the steady recovery of the US economy and the expected increase in interest rates, the high domestic zinc price has fallen back and continued to fall. Although it adapted to the rapid adjustment of its business ideas in the market, it is still affected by the overall business risk and financial risk. In 2016, due to the influence of such favorable factors as “capacity removal, inventory removal, deleveraging, cost reduction, and shortage compensation board,” the decline of zinc price eased and slowly rebounded. It can be seen from the forecast chart that although the actual value is low, the forecast value is above the healthy threshold line, and the actual value at the end of 2016 is much higher than the healthy threshold line, which shows the accuracy of the model. The actual value and forecast value of other prediction points are in the same healthy area, and the change direction of forecast value is consistent with the change direction of actual value in the next period, which further proves that Kalman filter model has good tracking and early warning of the risk of pledge financing.

The article "A Risk Decision-Making Model Based on Kalman Filter for Intellectual Property Pledge Financing" was published in 2022. Journal: Comput Intell Neurosci.

We take Carrier Holdings Co., Ltd. (stock code: 002072) as an example of risk-based enterprises. The enterprise is a cotton textile enterprise listed in 2006. Its main products are extra wide decorative fabric series, large and small jacquard fabric series, and so on. It is at high risk according to the risk classification criteria for pledge financing of the original samples. From the results of the forecast chart of the observation period, the enterprise is in the area of lower risk threshold for most of the time, and the overall situation is a high risk.

In 2014, affected by many factors, such as the downturn of domestic real economy and the rising price of factors of production, cotton textile enterprises had increased operating pressure causing domestic demand to slump continuously and its international market competitiveness to be declined significantly; in addition, the development of the textile industry has become more difficult. From individual observation points, the true values of the third and sixth phases are above the lower limit of the risk threshold, but the predicted values are in the severe risk area, and the subsequent fourth and fifth phases return to the severe risk area, thus confirming the accuracy of the decision-making results.

### 4.5. Total Discrimination Accuracy Analysis

The overall discriminatory accuracy analysis is shown in the following three areas:

1. Overall prediction accuracy analysis. Any risk decision-making model has its limitations or neglected influencing factors. Therefore, there is no perfect model which achieves 100% prediction accuracy. Prediction accuracy refers to the goodness or disadvantage of the fitting degree between the predicted value and the actual value produced by the prediction model, which reflects the fitting degree of the prediction model, and is also an important index to judge whether the prediction method has applicability. According to the test results, the average error between the predicted value and the real value of the seven-period semiannual reports is 8.5%, and the average error of the model in the last period is only 5.1%. Accordingly, the prediction accuracy of the model is high and the prediction effect is good.
2. Analysis of the results of risk-based test samples. From the predicted value calculated by the dynamic model of Kalman filter, if the last stage of the whole sample is risk-based, and 93% of the test samples in the sixth period are correctly predicted before the crisis occurs, that is, before the risk situation appears at the end of 2016, they have already fallen below the threshold of mild crisis or entered the area of high risk, and 93% of the samples have the mild financing risk two times in advance.
3. Analysis of the results of healthy-type test samples. From the predicted results of healthy samples, the predicted values of most healthy enterprises are above the warning line of mild-risk threshold. The predicted values of individual samples have temporarily deviated from the normal values at a certain point, but the dynamic model then corrects the situation in time. Even if they belong to mild-risk area, the predicted values of some healthy enterprises also deviate from the normal values, which means they are slightly below the warning line and are at a temporary mild risk. The results of 112 groups of dynamic data from 16 healthy enterprises showed that the recognition accuracy of healthy samples in the sixth period was 93.75% and the overall recognition accuracy was 87.5%.

The article "A Risk Decision-Making Model Based on Kalman Filter for Intellectual Property Pledge Financing" was published in 2022. Journal: Comput Intell Neurosci.

This paper further classifies the errors in classification recognition: class A and class B errors. When a risky financing enterprise is misjudged as a healthy enterprise, this is called class A error. If it is correctly identified, it is considered to be sensitive. Conversely, when a healthy enterprise is misjudged as a risky enterprise, this is called class B error. If it is correctly identified, it is considered to be specific. No matter what kind of mistake occurs, it may lead to wrong decision-making and cause serious losses. The accuracy of decision-making model in identifying risk categories is shown in Table 5.

According to the results in Table 5, the Kalman filter model has a high comprehensive judgment rate, which shows that the Kalman filter model has good robustness and prediction ability. The rate of misjudging a risky company as a healthy enterprise is 9.4%, the rate of misjudging a healthy company as a risky company is 12.5%, and the overall accuracy of the model is 89.1%. Among them, the rate of risky enterprises misjudged as healthy ones is lower than that of healthy enterprises misjudged as risky ones, which can further reduce the risk of pledge financing.

In addition, the results also illustrate that the risk criteria for IP pledge financing are likely to be more stringent than those of other financing ways. For banks and other lending institutions, it is necessary to change the previous cautious attitude towards IP pledge financing business.

## 5. Conclusion

Dynamic prediction can provide sufficient evidence for financing risk decision-making and reduce financing decision risk. In this paper, we established the pledge financing risk decision-making model based on Kalman filter, because of cumulative and time-varying characteristics of financing risks, and extracted the key variables affecting financing risk by principal component analysis method. Listed SMEs are tested and analyzed, and we found the following: (1) The average error between the predicted and the real values is 8.5%, so the model has higher fitting precision. (2) The rate of a risky company wrongly judged to be a healthy company is 9.4%. Conversely, the rate is 12.5% for a healthy company wrongly judged to be a risky company. The overall recognition accuracy of the model is 89.1%. (3) The risk decision-making model has high discriminant accuracy and can provide evidence to risk decision-making.

In this paper, we only established the pledge risk decision-making model based on Kalman filter. As we all know, the risk of IP pledge is a very complex problem. In future research, we will explore the establishment of a risk decision-making model based on combination of Kalman filter and neural network, so as to further improve the accuracy and effectiveness of the risk decision-making model.

## Figures and Tables

**Figure 1:** Some of the predictive value curves of testing the financing risk.

**Table 1:** Early-warning index system.

Type	Code	Indicator name
Debt paying ability	*X*_1_	Current ratio
	*X*_2_	Quick ratio
	*X*_3_	Asset-liability ratio
	*X*_4_	Cash ratio
	*X*_5_	Cash-maturity debt ratio
Cash flow	*X*_6_	Operating income to sales cash ratio
	*X*_7_	Operating income to net cash ratio
	*X*_8_	Cash operation index
Financial performance	*X*_9_	Return on equity
	*X*_10_	Profit on asset
	*X*_11_	Net profit on asset
	*X*_12_	Sales of net profit margin
Innovation capability	*X*_13_	Retained earnings on asset
	*X*_14_	R&D-revenue ratio
	*X*_15_	Number of bachelor degrees or above in staff
Asset operation	*X*_16_	Inventory turnover
	*X*_17_	Receivable turnover
	*X*_18_	Asset turnover
Growth ability	*X*_19_	Net profit growth ratio
	*X*_20_	Revenue growth ratio
	*X*_21_	Net asset growth ratio

The article "A Risk Decision-Making Model Based on Kalman Filter for Intellectual Property Pledge Financing" was published in 2022. Journal: Comput Intell Neurosci.

**Table 2:** Total variance explained.

Component	Initial eigenvalue			Extraction sums of squared loadings		
	Total	% of variance	Cumulative %	Total	% of variance	Cumulative %
1	4.221	20.102	20.102	4.221	20.102	20.102
2	2.996	14.268	34.370	2.996	14.268	34.370
3	1.693	8.063	42.433	1.693	8.063	42.433
4	1.340	6.380	48.813	1.340	6.380	48.813
5	1.304	6.208	55.021	1.304	6.208	55.021
6	1.162	5.534	60.555	1.162	5.534	60.555
7	1.045	4.976	65.532	1.045	4.976	65.532
8	0.998	4.753	70.285	0.998	4.753	70.285
9	0.891	4.244	74.529	0.891	4.244	74.529
10	0.848	4.039	78.568	0.848	4.039	78.568
11	0.819	3.902	82.470	0.819	3.902	82.470
12	0.754	3.593	86.062	0.754	3.593	86.062
13	0.708	3.372	89.434	0.708	3.372	89.434
14	0.572	2.722	92.156	0.572	2.722	92.156
15	0.477	2.274	94.430	0.477	2.274	94.430
16	0.442	2.105	96.535			
17	0.348	1.655	98.190			
18	0.302	1.436	99.626			
19	0.063	0.299	99.925			
20	0.008	0.040	99.965			
21	0.007	0.035	100.000			

**Table 3:** Coefficient matrix.

Component															
	1	2	3	4	5	6	7	8	9	10	11	12	13	14	15
*X*_1_	0.530	−0.798	0.193	0.012	−0.094	−0.051	−0.067	0.059	−0.035	−0.025	−0.007	−0.054	−0.027	−0.011	−0.033
*X*_2_	0.546	−0.791	0.206	−0.014	−0.060	−0.035	−0.045	0.087	−0.048	−0.015	0.022	−0.057	−0.009	0.015	−0.003
*X*_3_	−0.676	0.198	0.216	0.166	0.131	−0.137	−0.075	0.040	−0.010	0.047	0.260	−0.245	0.155	0.070	0.139
*X*_4_	0.515	−0.755	0.251	−0.013	−0.054	−0.040	−0.035	0.131	−0.040	0.026	0.047	−0.060	0.012	0.024	0.038
*X*_5_	0.186	0.086	−0.127	−0.147	0.481	0.188	0.089	0.529	−0.301	−0.011	0.482	0.047	0.134	−0.043	−0.085
*X*_6_	−0.032	0.022	0.271	0.164	0.497	−0.391	0.419	0.200	0.102	0.049	−0.428	−0.037	0.160	−0.123	−0.169
*X*_7_	0.339	0.141	0.227	−0.563	0.065	0.274	0.192	−0.040	0.064	0.349	−0.192	−0.093	0.314	0.114	0.267
*X*_8_	0.078	0.063	0.303	−0.410	0.037	0.037	0.434	−0.128	0.378	−0.539	0.249	−0.048	−0.154	0.009	0.016
*X*_9_	0.700	0.381	−0.033	0.015	0.072	−0.155	−0.146	−0.223	−0.050	−0.016	0.072	−0.052	0.001	−0.048	0.048
*X*_10_	0.808	0.446	0.043	−0.021	0.025	−0.078	−0.078	−0.116	−0.100	−0.029	0.034	−0.026	0.056	−0.212	0.055
*X*_11_	0.844	0.397	−0.003	−0.017	0.023	−0.081	−0.071	−0.112	−0.089	−0.030	0.014	0.021	0.026	−0.201	0.065
*X*_12_	0.506	0.215	0.035	0.096	0.103	−0.571	−0.058	−0.078	0.045	−0.029	0.140	0.146	0.096	0.491	−0.063
*X*_13_	0.425	0.227	−0.273	−0.121	0.337	0.238	−0.045	0.221	−0.068	−0.047	−0.313	−0.029	−0.495	0.240	0.005
*X*_14_	0.196	−0.342	−0.258	0.142	0.305	0.344	0.109	−0.356	0.243	0.160	0.112	0.482	0.156	0.034	−0.123
*X*_15_	0.215	−0.217	−0.125	0.612	0.430	0.154	0.108	−0.210	0.134	−0.031	0.075	−0.318	−0.090	−0.089	0.214
*X*_16_	−0.142	0.124	0.596	0.193	0.230	0.181	−0.435	0.194	0.208	−0.122	−0.068	0.245	0.009	0.108	0.257
*X*_17_	−0.002	0.138	0.433	0.295	−0.176	0.153	0.505	−0.192	−0.457	0.177	0.096	0.064	−0.192	0.193	0.066
*X*_18_	0.084	0.359	0.728	0.102	−0.006	0.241	−0.161	−0.053	−0.051	0.008	−0.018	0.088	−0.072	−0.148	−0.316
*X*_19_	0.290	0.243	0.032	0.119	−0.260	−0.131	0.130	0.330	0.488	0.500	0.238	0.030	−0.276	−0.092	0.012
*X*_20_	0.430	0.276	−0.069	0.257	−0.246	0.419	−0.025	0.099	0.200	−0.075	−0.035	−0.390	0.269	0.243	−0.258
*X*_21_	0.301	0.177	−0.180	0.379	−0.408	0.069	0.269	0.364	−0.027	−0.311	−0.140	0.294	0.191	−0.050	0.192

The article "A Risk Decision-Making Model Based on Kalman Filter for Intellectual Property Pledge Financing" was published in 2022. Journal: Comput Intell Neurosci.

**Table 4:** The real values and the predictive values of sample companies.

Data	Real value	Predictive value	Real value	Predictive value	Real value	Predictive value
Company code	002114		002098		002450	
2013.12.31	0.1716	0.1716	0.0691	0.0691	0.1049	0.1049
2014.06.30	0.1013	0.1540	0.0365	0.0609	0.0616	0.0940
2014.12.31	0.2328	0.1994	0.0653	0.0600	0.0930	0.0882
2015.06.30	0.2366	0.2348	0.0303	0.0369	0.0529	0.0597
2015.12.31	0.1252	0.1608	0.0684	0.0565	0.1014	0.0857
2016.06.30	0.0667	0.0810	0.0413	0.0467	0.0619	0.0700
2016.12.31	0.1647	0.1286	0.0856	0.0752	0.0932	0.0858

Company code	002139		002020		002014	
2013.12.31	0.1037	0.1037	0.0930	0.0930	0.0936	0.0936
2014.06.30	0.0517	0.0907	0.0657	0.0862	0.0415	0.0806
2014.12.31	0.1030	0.0929	0.1001	0.0924	0.0914	0.0818
2015.06.30	0.0554	0.0641	0.0531	0.0636	0.0467	0.0546
2015.12.31	0.1097	0.0935	0.0834	0.0740	0.1006	0.0845
2016.06.30	0.0535	0.0663	0.0523	0.0578	0.0543	0.0648
2016.12.31	0.1096	0.0957	0.0839	0.0750	0.0978	0.0877

Company code	002072		002125		002260	
2013.12.31	−0.0388	−0.0388	0.0612	0.0612	0.1104	0.1104
2014.06.30	−0.1847	−0.0753	0.0112	0.0487	0.0094	0.0852
2014.12.31	0.0553	−0.0036	−0.0421	−0.0192	0.0933	0.0787
2015.06.30	−0.0402	−0.0198	0.0168	−0.0066	0.0299	0.0388
2015.12.31	−0.2683	−0.2051	0.0681	0.0466	0.0369	0.0298
2016.06.30	0.0675	−0.0284	0.0552	0.0605	0.0318	0.0272
2016.12.31	0.0032	0.0136	0.0491	0.0567	−0.0286	−0.0168

Company code	002392		002571		002115	
2013.12.31	0.0578	0.0578	0.0607	0.0607	−0.0064	−0.0064
2014.06.30	0.0276	0.0502	0.0214	0.0509	−0.1934	−0.0531
2014.12.31	0.0399	0.0396	0.0386	0.0378	0.0500	−0.0051
2015.06.30	0.0131	0.0170	0.0122	0.0153	0.0375	0.0325
2015.12.31	0.0071	0.0050	−0.0341	−0.0266	0.0700	0.0688
2016.06.30	0.0125	0.0071	−0.0395	−0.0447	−0.0429	−0.0069
2016.12.31	0.0515	0.0398	0.0913	0.0524	0.0489	0.0262

The article "A Risk Decision-Making Model Based on Kalman Filter for Intellectual Property Pledge Financing" was published in 2022. Journal: Comput Intell Neurosci.

**Table 5:** Recognition accuracy of Kalman filter model.

Date	Class A error ratio (%)	Sensitivity (%)	Class B error ratio (%)	Specificity (%)	Recognition accuracy (%)
2016.12	6.25	93.75	6.25	93.75	93.75
2016.06	12.5	87.5	6.25	93.75	90.6
2015.12	6.25	93.75	12.5	87.5	90.6
2015.06	6.25	93.75	18.75	81.25	87.5
2014.12	12.5	87.5	12.5	87.5	87.5
2014–06	12.5	87.5	18.75	81.25	84.3

## Data Availability

The data used to support the findings of this study are available from the corresponding author upon request.
